# Elevated serum levels of Chromogranin A in hepatocellular carcinoma

**DOI:** 10.1186/1471-2482-12-S1-S7

**Published:** 2012-11-15

**Authors:** Antonio Biondi, Giulia Malaguarnera, Marco Vacante, Massimiliano Berretta, Velia D’Agata, Michele Malaguarnera, Francesco Basile, Filippo Drago, Gaetano Bertino

**Affiliations:** 1 Department of General Surgery, Section of General Surgery and Oncology, Vittorio Emanuele Hospital, Via Plebiscito 628 University of Catania, 95123 Catania, Italy; 2 International PhD programme in Neuropharmacology, University of Catania, Italy; 3 Department of Senescence, Urological and Neurological Sciences, Cannizzaro Hospital Via Messina 829, 95125, University of Catania, Italy; 4 Department of Medical Oncology, National Cancer Institute, Aviano [PN] Italy, Via Franco Gallini 2, 33081 Aviano [PN], Italy; 5 Department of Biomedical Sciences, Via S. Sofia, 87, 95123, University of Catania, Italy; 6 Department of Medical and Pediatric Sciences Via S. Sofia, 87, 95123, University of Catania, Italy

## Abstract

**Background:**

During the past three decades, the incidence of hepatocellular carcinoma in the United States has tripled. The neuroendocrine character has been observed in some tumor cells within some hepatocellular carcinoma nodules and elevated serum chromogranin A also been reported in patients with hepatocellular carcinoma. The aim of this work was to investigate the role of serum concentration of chromogranin A in patients with hepatocellular carcinoma at different stages.

**Methods:**

The study population consisted of 96 patients (63 males and 33 females age range 52-84) at their first hospital admission for hepatocellular carcinoma. The control group consisted of 35 volunteers (20 males and 15 females age range 50-80). The hepatocellular carcinoma patients were stratified according the Barcelona-Clinic Liver Cancer classification. Venous blood samples were collected before treatment from each patients before surgery, centrifuged to obtain serum samples and stored at -80° C until assayed.

**Results:**

The chromogranin A serum levels were elevated (> 100 ng/ml) in 72/96 patients with hepatocellular carcinoma. The serum levels of chromogranin A were significantly correlated (p<0.05) with alpha-fetoprotein. In comparison with controls, the hepatocellular carcinoma patients showed a significant increase (p<0.001) vs controls. The chromogranin A levels in the Barcelona staging of hepatocellular carcinoma was higher in stage D compared to stage C (p<0.01), to stage B (p<0.001), and to stage A (p<0.001).

**Conclusions:**

Molecular markers, such as chromogranin A, could be very useful tools for hepatocellular carcinoma diagnosis. However the molecular classification should be incorporated into a staging scheme, which effectively separated patients into groups with homogeneous prognosis and response to treatment, and thus serves to aid in the selection of appropriate therapy.

## Background

During the past three decades, the incidence of hepatocellular carcinoma (HCC) in the United States has tripled with an annual increase of 4.5% [1]. Two diagnostic tests are routinely used to detect HCC in clinical practice: serum α-fetoprotein (AFP) and ultrasonography (US). AFP is a glycoprotein, expressed during the early stages of fetal liver development by the endodermal cells of the visceral yolk sac, in the patients with testis cancer and during hepatocarcinogenesis. The sensitivity of AFP as a diagnostic tool is restricted by the existence of non-AFP-secreting tumors [2-5]. The reliability of ultrasonographic diagnosis depends on a range of factors, including the expertise of the operator, the sophistication of the equipment and the size and nature of the tumor. HCC commonly exhibits histological polymorphism even within a single nodule. The neuroendocrine character has been observed in some tumor cells within some HCC nodules and elevated serum chromogranin A (CgA) also been reported in patients with HCC [6,7]. CgA is a member of the granin family of acidic secretory glycoproteins that are expressed in all endocrine and neuroendocrine cells, in various autoimmune disease, and correlated with the use of various drugs, such as proton pump inhibitors. CgA has been identified in numerous variety of tumors, including bronchial [8], prostate [9], pancreatic and gastrointestinal cancer [10,11]. The aim of this work was to investigate the role of serum concentration of CgA in patients with HCC at different stages.

## Methods

The study population consisted of 96 patients [63 males and 33 females age range 52-84] at their first hospital admission for HCC. The control group consisted of 35 volunteers [20 males and 15 females age range 50-80]. The HCC patients were stratified according the Barcelona-Clinic Liver Cancer classification (BCLC) [12-14]. The BCLC staging classification links the stage of the disease to a specific treatment strategy. The BCLC uses variables related to tumour stage, liver functional status, physical status, and cancer-related symptoms, thus linking the four stages. The patients were recruited in a five years period (1^st^ January 2002- 31^st^ December 2006) and their demographics and clinical characteristics are shown in table 1. Venous blood samples were collected before treatment from each patients before surgery, centrifuged to obtain serum samples and stored at -80 °C until assayed. Clinical chemistry tests were performed in the medical centre laboratory using standard methods. Fasting blood samples were taken at enrolment of the participants. Hepatitis B surface antigen (HbsAg) and its antibody (HbcAb) and antibody to delta antigen (anti-HDV) were all determined by enzyme immunoassay (Abbott Laboratories, North Chicago, IL). Antibody to hepatitis C virus (anti-HCV) was assayed by a second-generation enzyme-linked immunoassay (ELISA, Ortho Diagnostixc Systems-Raritan, NJ). Specific investigations included abdominal US and triphasic spiral computerized tomography or magnetic resonance (MR). A US-guided liver biopsy was performer using a 18–21 range needle to sample both liver parenchyma and focal lesion. A commercial solid phase two site immunoradiometric assay was used to detect serum CgA (CgA-RIA CT, CIS Biointernational ORIS Group, GIF-SUR-Yvette, France). AFP was tested by using commercially available immunometric assay (Architect AFP assay, Abbott Laboratories, North Chicago, IL, USA). All data are presented as mean ±S.D. Discrete and continuous variables were compared using either Student’s t-test or the Wilcoxon Mann–Whitney non-parametric test for unpaired data. Categorical variables were compared with either the Chi square test or the Fisher exact test when requested. The Spearman’s rank correlation coefficient test was used to test for unvaried relationships between variables. The applied tests were considered statistically significant at p<0.05 level. Data were analyzed using the statistical package SPSS for Windows 7.5 (SPSS Inc., Chicago, IL, USA).

**Table 1:** Demographic characteristics of subjects included in the study.

Parameter	Stage 0	Stage A	Stage B	Stage C	Stage D	Controls
Number	15	21	19	24	17	35

Male\Female	10\5	15\6	10\9	17\7	11\6	20\15

Smokers yes\no	12\3	16\5	15\4	16\8	10\7	18\17

Heart rate b\m	78±6	84±5	77±8	88 ± 7	94 ± 7	78 ± 10

Systolic Pressure mmHg	135±10	144±12	141±13	140±12	145±10	136±10

Diastolic Pressure mmHg	84±8	88±10	85±9	87±8	88±9	84±7

HCV	6	7	9	10	10	-

HBV	5	8	8	8	4	-

Alcool	4	6	2	6	3	-

## Results and discussion

The CgA serum levels were elevated (> 100 ng/ml) in 72/96 patients with HCC (Table 2). No significant differences were found between males and females in either of the groups. The serum levels of CgA were significantly correlated (p<0.05) with AFP. In comparison with controls, the HCC patients showed a significant increase (p<0.001) compared to controls. The CgA levels in the Barcelona staging of HCC was higher in stage D compared to stage C (p<0.01), to stage B (p<0.001), and to stage A (p<0.001). The most frequent site of neuroendocrine tumours is the gastrointestinal tract, accounting for approximately 70% [15] of the total neuroendocrine tumours in the body [16,17]. Neuroendocrine tumours frequently metastasize to the liver, but the liver itself seldom is the site of a primary tumour [18-20]. The etiology and histogenesis of hepatic neuroendocrine tumours have remained elusive and controversial [21]. Proposed theories on the origin of neuroendocrine cells, that give rise to primary hepatic neuroendocrine tumours, include ectopic neuroendocrine cells of pancreatic or adrenal origin, neuroendocrine cells from within the intraepatic biliary tree or from neuroendocrine-programmed ectoblasts [22]. The origin of neuroendocrine components in HCC can be explained by the neuroendocrine cells existing in the original HCC tumour as one of the histological components; or the occurrence of phenotypic change and/ or differentiation of HCC cells; a differentiation from hepatic stem cells [23]. HCC is a complex neoplasm, in most cases on a background of preneoplastic damaged liver. An hypothesis describes a step-by-step process through which external stimuli could induce genetic alterations in mature hepatocytes leading to cell death and cellular proliferation. In the progression of chronic inflammation to fibrosis and cirrhosis, the up-regulation of mitogenic pathways leads to the production of monoclonal populations. These populations harbour dysplastic hepatocytes as a result of altered gene expression and telomerase erosions. Thus, molecular markers, such as CgA, could be very useful tools for HCC diagnosis [24]. However the molecular classification should be incorporated into a staging scheme, which effectively separated patients into groups with homogeneous prognosis and response to treatment, and thus serves to aid in the selection of appropriate therapy.

**Table 2:** AFP and CgA levels of the subjects included in the study according to the BCLC classification

	α-Fetoprotein	CgA
Controls	3.8 ± 1.2	73 ± 10

Stage 0	16 ±4	96 ± 6

Stage A	24 ± 6	102 ± 10

Stage B	36 ± 8	125 ± 12

Stage C	74 ± 24	145 ± 96

Stage D	128 ± 36	210 ± 110

## List of abbreviations

HCC: Hepatocellular Carcinoma; AFP: α-fetoprotein; US: Ultrasonography; CgA: Chromogranin A; BCLC: Barcelona-Clinic Liver Cancer; MR: Magnetic Resonance.

## Competing interests

The authors declare that they have no competing interests.

## Authors’ contributions

AB, GM: conception and design, interpretation of data, drafting the manuscript, given final approval of the version to be published; MV, MB, VDA, MM: acquisition of data, drafting the manuscript, given final approval of the version to be published; FB, FD, GB: critical revision, given final approval of the version to be published.
